# Comparison of Improved Surgical Eight-Step Handwashing Combined with ATP Fluorescence in Detecting the Infection Rate at the Site of Seven-Step Surgical Handwashing and 30-Day Orthopaedic Surgery: A Randomized Study

This article has been retracted.

**DOI:** 10.1155/2022/3123565

**Published:** 2022-07-19

**Authors:** Xiong Chen, Tao Wang, Qinglian Li, Lixia Cheng, Zhimin Xie, Jianping Xu, Dejian Yang

**Affiliations:** ^1^Department of Operating Room, Xianyou County General Hospital, Putian 351200, China; ^2^Department of Orthopedics, Beijing Jishuitan Hospital, Beijing 100035, China; ^3^Department of Orthopedics, Putian Medical District, The 900th Hospital of Joint Logistic Support Force, PLA, Putian 351100, China

## Abstract

**Objectives:**

To compare the effects of two hand cleaning schemes on the prevention of surgical site infection in routine orthopaedic surgery. Compared with the standard surgical seven-step washing technique and detected by ATP fluorescence method, the handwashing effects of the improved surgical eight-step washing technique and the standard surgical seven-step washing technique were compared, so as to provide a basis for eliminating the handwashing blind area of the surgical seven step washing technique and improving the surgical handwashing method.

**Methods:**

A total of 800 consecutive patients who underwent clean and clean-contaminated orthopaedic surgery between January 1, 2020 and December 31, 2020. Twenty orthopaedic doctors in the operating room of our research team were randomly divided into the improved eight-step washing technique group (improved group) and the traditional seven-step washing technique group (traditional group), with 10 people in each group. Each person was randomly sampled 40 times, 400 people in each group, a total of 800 people, and completed by stages in 12 months. *Main Outcome Measures*. The infection rate of surgical site 30 days after operation was the primary end point. The qualified rate of fingertip culture was combined with ATP fluorescence in the two groups and three new culture areas in the two groups: the lateral edge of the palm, the medial edge of the palm, and the nail groove of the middle finger and the nail root were secondary end points.

**Results:**

The 2 protocols were comparable in regard to surgical site infection risk factors. The infection rate of surgical site in the traditional group was 10 cases (2.50%) in 400 cases and 0 cases (0%) in the improved group. Three culture areas were added: the qualified rate of lateral edge of palm, medial edge of palm, and nail groove and nail root of middle finger, and the nosocomial infection rate of surgical incision between the two groups was statistically significant (*P* < 0.05). There was no significant difference in the qualified rate of fingertip culture (*P* > 0.05). The handwashing scheme in this study meets the recommended duration of hand disinfection and has good tolerance, and the skin dryness and skin irritation after using aqueous solution are similar.

**Conclusions:**

The improved surgical eight-step washing technique combined with ATP fluorescence detection is helpful to eliminate the “blind area” of handwashing. It is also necessary to add three training areas. Handwashing and training are more scientific, rigorous, and effective. They are effective in reducing orthopaedic surgical infection and have application value. They can safely replace the traditional surgical seven-step washing technique, which is worthy of clinical promotion.

## 1. Background

Due to China's large population, limited medical resources, large-scale medical institutions, dense patients, and heavy workload of medical staff, medical staff often ignore hand hygiene, resulting in pollution and hospital infection; Hand is an important way to spread the sense of hospital. Surgical site infection prolongs hospital stay, is one of the main causes of incidence rate, and is also the source of high medical expenses [1]. Hand hygiene is the simplest, most direct, and effective measure to prevent nosocomial infection, and it is also one of the most important tasks in nosocomial infection management [2, 3]. Few clinical studies have compared the risk of infection in orthopaedic surgery after different cleaning methods. Orthopaedic surgery has more open fractures, and the incision is polluted incision, which is more prone to infection, because most of them have built-in objects, and orthopaedic doctors' fingers are more prone to occupational exposure, especially the fingertips of index fingers and nail grooves are easily pierced by Kirschner wire tips, broken ends of bones, and other accidents, resulting in occupational exposure. The nosocomial infection rate of surgical incision is high. Therefore, orthopaedic doctors have higher requirements for handwashing. Handwashing is the most economical and effective means of prevention and control. The standard surgical seven-step washing technique is improved compared with the previous six-step washing technique, and the technology has become mature, but there are still “blind areas” where the cleaning is not in place. It is more necessary to sample and cultivate the “blind areas” after handwashing, and there is a lack of relatively objective evaluation criteria for washing to 10 cm above the elbow and applying disinfectant to 6 cm above the elbow. The current standard surgical seven-step washing technique has three handwashing blind areas and training blind areas. The seven-step washing technique lacks relatively objective evaluation criteria to wash hands to 10 cm above the elbow and apply disinfectant to 6 cm above the elbow, which needs to be further improved.

## 2. Introduction

In this study, three handwashing blind areas and training blind areas existed in the standard surgical seven-step washing technique were improved. While using the standard fingertip sampling culture, the sampling culture of hand-washing blind areas was increased. The qualified rate of handwashing and the nosocomial infection rate of orthopaedic surgical incision were compared between the two groups.

## 3. Data and Methods

### 3.1. Clinical Data

From January to December 2020, the handwashing environment and other conditions were the same. 20 orthopaedic doctors in the operating room environment were selected and randomly divided into the improved group and the traditional group, with 10 people in each group. Each person was randomly sampled 40 times, with 400 people in each group, a total of 800 people. They were completed in stages in 12 months. Combined with ATP fluorescence method, the qualified rates of three new culture areas in the two groups: the lateral edge of the palm, the medial edge of the palm, and the nail groove and nail root of the middle finger, were detected and compared, and the qualified rates of fingertip culture and the nosocomial infection rate of the incision after operation were compared between the two groups. The sampling work was completed by the members of this study in stages.

### 3.2. Research Method

#### 3.2.1. Handwashing Method

① The traditional group used standard surgical seven-step washing to wash hands. ② The improved group used the improved surgical eight-step washing technique and washed the arm for the first time: washing hands to 5 horizontal fingers on the elbow was the objective standard. Wash your arms for the second time: wash your hands to 4 horizontal fingers on the elbow as the objective standard, and apply disinfectant to 3 horizontal fingers on the index finger, middle finger, and ring finger as the objective standard. The first seven steps are the same as above. Step 8: similar to step 6, close your fingers together and put them on the other hand. There are three blind areas: the outer edge of the palm, the inner edge of the palm, and the nail groove and the nail root, which are carried out alternately.

#### 3.2.2. Sampling Method

Before and after handwashing, each subject took 4 samples from four culture areas, including conventional fingertips, and three new culture areas: the outer edge of the palm, the inner edge of the palm, and the nail groove of the middle finger and the root of the nail. Spin and smear the cotton swab of the bacterial culture tube at the above four sampling places twice and submit it for inspection; biological detection method: take the samples stored in PBS and shake them sufficiently to make the microorganisms on the cotton swab dissolve in PBS as much as possible. After the Petri dish is numbered, add 0.5 ml of the sample into the Petri dish, spread it evenly with a sterile l rod, and make 3 copies of each sample. After all smearing and culture, put it into 37°C incubator for 72 hours. Record the number of growing colonies and calculate the average value as the test result. The control adopts PBS solution control and empty Petri dish control. The positive control of Escherichia coli is added to the Petri dish. It is cultured at 37°C for 72 hours with the sample for observation and detected by ATP fluorescence method. Observe and record the results of finger improved surgical eight-step handwashing combined with ATP fluorescence detection and bacterial culture+drug sensitivity test after surgical washing manipulation.

#### 3.2.3. Interventions

Calculation formula of biological monitoring quantity is as follows: total bacteria (CFU/cm^2^) = plate colony × dilution multiple/sampling area (cm^2^). The ATP fluorescence test of the operator is negative, and the bacterial culture ≤ 5 CFU/cm^2^ is qualified. The infection rate of the operation site was calculated when the patient had no infection at the operation site within 30 days after the operation, which was negative and positive. 30 days after operation, the infection rate of operation site in the two groups was the primary end point. The qualified rate of fingertip culture in the two groups and three new culture areas in the two groups: the lateral edge of the palm, the medial edge of the palm, and the nail groove of the middle finger and the nail root were detected by ATP fluorescence method. The qualified rate of culture after operation was the secondary end point. The SPSS23 0 statistical software was used for data analysis. The normal measurement data is expressed by “mean ± SD,” and the counting data is expressed by the number of cases or percentage.

## 4. Result

### 4.1. Bioassay Results before and after Handwashing

Before handwashing, the number of bacteria in the hands of orthopaedic doctors in the traditional group was 29.32~593.32 CFU/cm^2,^ respectively, and the detection result of ATP fluorescence method was positive. Before handwashing, the number of bacteria in the hands of orthopaedic doctors in the improved group was 28.32~596.32 CFU/cm^2^, respectively, and the detection result of ATP fluorescence method was positive. The hand hygiene of the two groups before handwashing was similar. After handwashing, the total number of bacteria in the hands of orthopaedic doctors in the traditional group is 1.32~62.67 CFU/cm^2^, respectively, which indicates that careful handwashing with flowing water and hand sanitizer can significantly reduce the amount of bacteria in the hands, and as long as they are cleaned according to the normal operation, they can basically meet the hygienic standard. In the improved group, the total number of bacteria in the hands of orthopaedic doctors was 1.32~32.67 CFU/cm^2^, respectively, indicating that the amount of bacteria in the hands can be greatly reduced by carefully washing hands with improved step washing method with flowing water and hand sanitizer, and the hygienic standard can be reached as long as they are cleaned according to the normal operation. The infection rate between the two groups was statistically significant.

### 4.2. Pass Rate after Handwashing

From January 2020 to December 2020, according to the biological monitoring results after handwashing by orthopaedic doctors, the qualified rate of conventional fingertips, lateral edge of palm, medial edge of palm and nail groove and nail root of middle finger were 97%, 91%, 90% and 92%, respectively. In the improved group, the qualified rates of conventional fingertip, lateral edge of palm, medial edge of palm, and nail groove and root of middle finger were 98%, 97%, 98%, and 99%, respectively. There was no significant difference in the qualified rate of fingertip samples between the two groups (*P* > 0.05). There were significant differences in the samples of the lateral edge of the palm, the medial edge of the palm, and the nail groove of the middle finger and the nail root (*P* < 0.05) (Table 1).

### 4.3. Biological Monitoring Results after Handwashing

After 800 orthopaedic doctors washed their hands, the number of samples in the traditional group was 400, and the incision infection rate was 2.5%. The number of samples in the improved group was 400, and the incision infection rate was 0%. The difference was statistically significant (*P* < 0.05) (Table 2).

See Table 1 for the comparison of the qualified rate of handwashing between the two groups.

See Table 2 for the comparison of infection rate of handwashing surgical incision between the two groups.

## 5. Discussion

In the 19th century, Semmelweis first noted the link between hospital-acquired diseases and hand hygiene [4]. Nosocomial infection places a heavy burden on patients and health care providers and economically affects health care institutions [5]. Hand is the main carrier of transmitting bacteria, viruses, and microorganisms. Bacteria carried by surgeons' hands or arms are the culprit of surgical incision infection and one of the most important factors. Surgical cleaning and surgical handwashing disinfection are effective methods to prevent handwashing. Hospital surgical wound infection is an important measure to prevent infection. Hand hygiene has always been an important part of perioperative practice. Effective handwashing is one of the most simple and easy means, an important measure to prevent exogenous hospital feeling, and an effective means of two-way protection between patients and medical staff. The sense of hospital has brought great economic impact to medical institutions. However, studies [6] have proved that the audit cycle can improve the efficiency of surgical handwashing. Among all tested compounds, the local skin microflora was significantly lower than that before scrubbing at two time points after scrubbing and operation [7]. Research [8] shows that handwashing feedback video monitoring is an effective tool to measure hand hygiene and improve compliance. Surgical site infection (SSI) remains a major problem for patients and medical systems. Paying attention to nursing and standardized quality measures continue to promote the improvement of surgical sterility, but there are still some disputes in the field of surgical hand disinfection [9]. It has been reported [10, 11] that the preoperative surgical hand disinfection scheme of hand is related to surgical wound infection (SSI). Preoperative handwashing is essential to prevent surgical site infection (SSI) [12]. Careful surgical scrubbing can reduce the number of bacteria on the skin, but it cannot completely eliminate bacteria. There are temporary microorganisms left on the hands after surgery. Studies [13] have proved that two-layer wound closure during surgical handwashing is not only an effective barrier to prevent microbial transmission, but also an effective barrier to protect surgeons. Handwashing is a necessary measure to prevent nosocomial infection [14]. Studies [15–17] have shown that effective hand hygiene, such as effective handwashing and hand disinfection, is the basis for slowing down the spread of COVID-19. The novel coronavirus pneumonia is being studied and popularized by studying the [18] medical staff's handwashing and hand disinfection. After hand disinfection, nails coated with conditioner or mixed varnish have a similar risk of pathogenic microorganisms as natural nails. Lasting regular nail polish will increase the risk of hand disinfection ineffective [19]. Clinical application of handwashing brush although the skin is common all over the world, the feeling, appearance, and integrity of the skin are obvious. It even causes serious damage. Pittet et al. [20] confirmed that after the pathogen is discharged from the infection source, it needs five consecutive steps to colonize or infect the new host. The seven-step washing technique includes the outer edge of the palm, the inner edge of the palm, and the nail groove of the middle finger and the root of the nail. There are “blind areas” in the seven-step washing technique. There are many wrinkled skin, and it is relatively difficult to clean and disinfect. Young medical personnel, especially interns, are mostly limited to textbooks, and their handwashing is easy to miss or insufficient, resulting in infection at the surgical site. ATP bioluminescence is a sensitive and rapid method for evaluating the quality of end cleaning. We emphasize the value of using quantitative methods to monitor the cleanliness of hospital environment [21]. Studies have shown that ATP biological fluorescence method has a certain correlation with the traditional bacterial culture method, can better reflect the cleaning status of hands, can help measure the sanitary quality of hospital surface, and can be used as a useful agent of microbial pollution [22]. By providing rapid feedback, ATP analysis helps to raise the awareness of operators and allows immediate action in case of emergency [23]. The research shows that ATP biological fluorescence detection method can provide an objective and real-time analysis method and effectively reduce the nosocomial infection rate [24–27]. After the application of ATP biological fluorescence on-site monitoring method, the hand hygiene compliance of all kinds of personnel in the operating room is higher than that before the application, and the qualified rate of hand hygiene is higher than that before the application, indicating that the hand hygiene compliance and qualified times of all kinds of personnel can be improved. Through regular on-site random sampling inspection, strengthen supervision and ensure the safety of patients and personnel. At the same time, formulate scientific, simple, and fast on-site hand hygiene monitoring standards, reduce the monitoring cost, eliminate the occurrence of nosocomial infection caused by poor hand disinfection effect, and improve the quality and image of medical services, which is expected to provide reference basis for on-site standardized management of hand hygiene. However, there is still a certain infection rate of surgical incision after rubbing and washing hands, especially in patients with orthopaedic surgery, surgical treatment, large incision surgery, long operation time, large intraoperative bleeding, and so on. It is easy to be infected and affect the treatment effect of infection in patients undergoing orthopaedic surgery. In serious cases, it will endanger the life of patients. Orthopaedic surgery has more open fractures, and the incision is polluted incision, which is more prone to infection, because most of them have built-in objects, and orthopaedic doctors' fingers are more prone to occupational exposure, especially the fingertips of index fingers and nail grooves are easily pierced by Kirschner wire tips, broken ends of bones, and other accidents, resulting in occupational exposure. The nosocomial infection rate of surgical incision is high. Therefore, orthopaedic doctors have higher requirements for handwashing.

This study focuses on orthopaedics with higher risk of implant infection, which requires higher and more rigorous surgical procedures. If it can reduce the infection of orthopaedic surgery, the improved eight-step washing technique is suitable for preoperative handwashing in orthopaedics and other surgeries with built-in objects, and it is also more suitable for preoperative handwashing in other surgeries. ATP fluorescence method and traditional bacterial culture method are effective and scientific. ATP fluorescence method is simpler than traditional bacterial culture method.

Therefore, this study selected a group of orthopaedic doctors as the research object. It was found that the two handwashing methods were handwashing and sampling according to the requirements of disinfection technical specifications. There was no significant difference in the qualified rate of fingertip samples (*P* > 0.05). It shows that the disinfection of fingertips by standard seven-step washing technique is qualified. However, there were three new culture areas: the lateral edge of the palm, the medial edge of the palm, and the nail groove and nail root of the middle finger. The difference of the infection rate of the surgical incision was statistically significant. The difference was statistically significant (*P* < 0.05). It shows that the seven-step washing technique has a “blind area.” The improved surgical eight-step washing technique combined with ATP fluorescence detection is helpful to eliminate the “blind area” of handwashing. It is also necessary to add three training areas. Handwashing and training are more scientific, rigorous, and effective. They are effective in reducing orthopaedic surgical infection and have application value. They are worthy of preoperative handwashing with built-in devices in clinical orthopaedics and are also more suitable for preoperative handwashing in other surgeries. In addition, orthopaedic doctors wear double gloves to prevent occupational exposure caused by accidental puncture of Kirschner wire tip and broken bone end, which is also worthy of promotion. Novel coronavirus pneumonia, which is now safe, more scientific, more rigorous, and effective, is also worth promoting in the new crown pneumonia epidemic. It can reduce cross infection, protect the patients who are fighting the epidemic, and protect the people in the isolated area. The eight-step washing technique is also worth promoting in the COVID-19.

## Figures and Tables

**Table 1:** Comparison of qualified rate of 4 samples of handwashing between two groups.

Group	Fingertip sample		Sample of lateral margin of palm		Sample of medial margin of palm		Nail groove and nail root samples of middle finger	
	Number of samples	Qualified rate (%)	Number of samples	Qualified rate (%)	Number of samples	Qualified rate (%)	Number of samples	Qualified rate (%)
Improvement group	400	98	400	97	400	98	400	99
Traditional group	400	97	400	91	400	90	400	92
*χ* ^2^	0.410		6.383		11.348		11.402	
*P*	>0.05		<0.05		<0.05		<0.05	

**Table 2:** Comparison of incision infection rate between two groups.

Group	Number of samples	Incision infection rate (%)
Improvement group	400	0
Traditional group	400	2.5
*χ* ^2^	5.063	
*P*	<0.05	

## Data Availability

The data used to support the findings of this study are available from the corresponding author upon request.
